# Proteomic Analyses Reveals the Mechanism of Acupotomy Intervention on the Treatment of Knee Osteoarthritis in Rabbits

**DOI:** 10.1155/2022/5698387

**Published:** 2022-11-17

**Authors:** Jing Liu, Weiquan Zeng, Qiaoxuan Lin, Rongqiong Dai, Liming Lu, Zexing Guo, Xiaowen Lian, Xigui Pan, Hong Liu, Zhong-Biao Xiu

**Affiliations:** ^1^The Affiliated People's Hospital of Fujian University of Traditional Chinese Medicine, Fuzhou 350004, China; ^2^Rehabilitation Hospital Affiliated to Fujian University of Traditional Chinese Medicine, Fuzhou 350003, China; ^3^The Third People's Hospital of Fujian Province, Fuzhou 350122, China; ^4^Fujian University of Traditional Chinese Medicine, Fuzhou 350122, China; ^5^Key Laboratory of Orthopedics & Traumatology of Traditional Chinese Medicine and Rehabilitation Ministry of Education, Fujian University of TCM, Fuzhou 350122, China; ^6^Fujian Institute of Orthopaedics, Fuzhou, Fujian 350004, China

## Abstract

Acupotomy intervention (AI) is an available treatment for knee osteoarthritis (KOA) in China, which is a common health problem over the world. However, the underlying mechanism of AI on the KOA treatment is still unknown. To further understand the mechanism of acupotomy in treating KOA, the morphological observation and TMT proteomic analyses were conducted in rabbits. By using X-ray and MRI, we found that the space of the knee joint was bigger in AI than in KOA. Moreover, the chondrocytes were neatly arranged in AI but disordered in KOA. With proteomic analyses in chondrocytes, 68 differently accumulated proteins (DAPs) were identified in AI vs. KOA and DAPs related to energy metabolism and the TCA cycle were suggested to play a central role in response to AI. Furthermore, AIFM1 was proposed to be an important regulator in controlling the energy production in mitochondrial. Besides, FN1, VIM, COL12A1, COL14A1, MYBPH, and DPYSL3 were suggested to play crucial roles in AI for the treatment of KOA. Our study was systematically elucidating the regulation mechanism of acupotomy intervention in the treatment of KOA.

## 1. Introduction

Knee osteoarthritis (KOA) is a chronic degenerative disease mainly characterized by knee ligament relaxation, degeneration of knee cartilage, and peripheral muscle atrophy [1]. KOA is caused by wear and tear subsequently and leads to abnormal remodelling and joint failure [2]. During this process, a series of physiological and molecular changes in multiple tissues inside the joint were observed [3]. As Haartmans et al. (2021) pointed out that a group of molecules rather than one specific biomarker will provide the possible therapeutic targets for KOA [3]. Therefore, a systematic understanding of the proteomic changes in KOA development was required.

As the common methods of traditional Chinese medicine (TCM) used for the treatment of KOA, acupotomy intervention (AI) was widely used to relieve cartilage tissue pain and restore the movement of the knee joint [4]. In rabbits, acupotomy could alleviate cartilage deterioration by regulating the OPG/RANKL signaling pathway to inhibit subchondral bone resorption [5]. Similarly, Huang et al. (2020) reported that activating the PI3K/Akt signaling pathway to inhibit the chondrocyte apoptosis in KOA rabbits might be a possible mechanism of acupotomy in treating KOA [6]. Moreover, the GSK3 beta-cyclin D1-CDK6 pathway was also regarded as a responsible mechanism of acupotomy to alleviate cartilage degeneration in KOA rabbits [7]. However, the systematic change of acupotomy intervention in treating KOA is still unknown. In the present study, the morphological and proteomic changes in rabbits treated with KOA and AI were analyzed to investigate the underline mechanism of acupotomy intervention in treating KOA.

## 2. Materials and Methods

### 2.1. Ethics Statement

Animal experiments were strictly handled following the regulations on the use and ethics of animals promulgated by the Ministry of Science and Technology, P.R.C. in 2006. Rabbits were provided by the Shanghai Songlian Experimental Animal Co. LTD. (License No. SCXK (Shanghai) 2017-0008) with a certification of fitness (No. 20170008001679), and the Experimental Animal Center of the Fujian University of Traditional Chinese Medicine (License No. SYXK (Fujian) 2020-0003) was entrusted to raise the animal. The ethical approval for research involving animals was approved by the Animal Experiment Ethics Committee of the Fujian University of Traditional Chinese Medicine.

### 2.2. Reagents and Materials

New Zealand white rabbits were purchased from Shanghai Songlian Experimental Animal Co. Ltd. (License No. SCXK (Shanghai) 2017-0008).

The disposable acupotome was purchased from Jiangxi LaoZongYi Medical Instrument Co. Ltd. (Jiangxi, China). Protease inhibitor cocktail, urea, dithiothreitol, iodoacetamide, TEAB, trypsin, BCA staining kit, and Masson staining kit were purchased from Beijing Solarbio Technology Co. Ltd (Beijing, China). Polyvinylpyrrolidone, sodium pentobarbital, acetonitrile, and formic acid were purchased from Thermo Fisher Biotechnology Co. Ltd. (USA). Polymer gypsum was purchased from Shanxi Anxin Medical Technology Development Co. Ltd. (Shanxi, China), and common gypsum was purchased from Pujiang Jianyu Sanitary Materials Co. Ltd. (Shanghai, China). Surgical blades and related instruments were purchased from Shanghai Medical Devices Wholesale Department Co. Ltd. (Shanghai, China).

### 2.3. Animals and Study Design

Nine male New Zealand white rabbits (6 months old) weighing approximately 2.0 ± 0.5 kg were raised without limitations of food and water in separate cages with 50%–60% humidity and 20°C–25°C temperature. After acclimation for one week, rabbits were randomly divided into 3 groups including the blank control group (CK, *n* = 3), rabbits with knee osteoarthritis (KOA, *n* = 3), and KOA rabbits treated with acupotomy intervention (AI, *n* = 3).

### 2.4. KOA Induction and Acupotomy Intervention

The induction of KOA rabbits was performed following the methods described by Wang et al. (2019) [8]. As the KOA model was established for one week, three points located (on left hind leg) at the tendons of quadriceps femoris, vastus medialis, and vastus lateralis were selected as the fixed intervention points. Polyvinylpyrrolidone was used for routine disinfection on the intervention points for three times and the three intervention points located at the tendons of quadriceps femoris, vastus medialis, and vastus lateralis. After disinfection, the blade of the acupotome was vertically inserted into the skin and parallel to the longitudinal axis of the tendons. The local adhesion to the direction of tendons and bone connection was released by longitudinal dredging and transverse stripping. After the acupotomy intervention, we pressed the intervention points for 1 min. The acupotomy intervention was performed every 7 d for 4 weeks.

### 2.5. The Observation of Knee Joints by using X-Ray, MRI, and a Light Microscope

After KOA induction, the rabbits were anesthetized by intraperitoneal injection with 3% sodium pentobarbital solution (1.5 mL/kg). For X-ray examination, the anteroposterior radiographs were taken in the supine position with hip flexion at 30°, knee extension at 0°, hip abduction at 15°, and keeping the patella in right forward. The radiating tube was 110 mm away from the knee joint. The left hind leg was extended and placed in the decubitus position, while the right hind leg was bent at 70°, and the knee was bent at 45°. The parameters for X-ray examination were set as follows: tube voltage 50 kV, current 250 mA, exposure strength 32 mAs, and exposure time for 128 ms.

For MRI (MAGNETOM Prisma 3.0T, Siemens, Germeny) examination, the rabbits were kept in the supine position and the knee was adjusted to a valgus position with a fixed angle of 15°. The patella was kept at the center of the scanner. The parameters for MRI examination were set as follows: (1) T1-tse-cor (FOV:100 × 100 mm、ST:2 mm、TR:831 ms、TE:11 ms); (2) T2-tse-sag (FOV:100 × 100 mm、ST:2 mm、TR:6860 ms、TE:84 ms).

The histomorphological observation of femoral condyle cartilage in rabbits was performed with hematoxylin-eosin (HE) staining and safranin O-fast green staining using standard protocols (Solarbio, Beijing, China).

### 2.6. Protein Extraction

Tissues used for protein extraction were stripped from tibia. The complex tissues containing cartilage-subchondral bone were intercepted from the central weight-bearing area of the tibia. Then, the cartilage tissues were isolated from the cartilage-subchondral bone complex tissues and put into liquid nitrogen directly. The chondrocytes from each treatment were grinded by liquid nitrogen into cell powder and transferred to a 5 mL centrifuge tube. Four volumes of lysis buffer (8 M urea, 1% protease inhibitor cocktail) were added to the cell powder and sonication on ice three times by using a high intensity ultrasonic processor (Scientz, Ningbo, China). The mixture was centrifuged at 12,000 g at 4°C for 10 min. After that, the supernatant was collected and the protein concentration was measured with a BCA kit according to the manufacturer's instructions (Figure 1). Each group had three replicates.

### 2.7. TMT Labeling and LC-MS/MS Analysis

The protein solution was reduced with 5 mM dithiothreitol (DTT) at 56°C for 30 min and alkylated with 11 mM iodoacetamide in darkness at room temperature for 15 min. After that, the mixed solution was diluted with TEAB (100 mM) to reduce the urea concentration (less than 2 M). Then, the protein in the mixed solution was digested overnight by trypsin with a mass ratio (trypsin to protein) of 1 : 50 and for another 4 h with a mass ratio (trypsin to protein) of 1 : 100. After digestion, peptide was desalted and vacuum-dried. Peptide was redissolved in 0.5 M TEAB and labeled by TMT following the manufacturer's instruction.

The digested peptides were fractionated into 60 fractions by using a pH reverse-phase C18 column (5 *μ*m, 10 mm, 250 mm, Betasil C18, Thermo Fisher Scientific, USA) with acetonitrile (pH 9.0) from 8% to 32% over 60 min. Then, the 60 fractions were divided into 6 fractions and vacuum-dried.

The tryptic peptides were dissolved in 0.1% formic acid (solution A) and loaded onto a home-madereversed-phase analytical column (15 cm length, 75 *μ*m i.d.). The settings for UPLC (EASY-nLC 1000 UPLC, Thermo Fisher Scientific, USA) were shown as follows: (1) gradient increase of solution B (0.1% formic acid in 98% acetonitrile) from 6% to 23% for 26 min; (2) 23% to 35% of solution B in 8 min; (3) 35% to 80% of solution B in 3 min; (4) kept at 80% for 3 min. The flow rate was kept at 400 nL·min-1, the electrospray voltage was 2.0 kV, the m/*z* ranged from 350 to 1800, and the resolution of the orbitrap was 70,000. Peptides were selected for MS/MS (Thermo Fisher Scientific, USA) using NCE setting as 28, and the resolution of the orbitrap was 17,500. Automatic gain control was 5E4, and fixed first mass was 100 m/*z*. The MS/MS data were processed by using the MaxQuant search engine (v.1.5.2.8). Tandem mass spectra were searched against the human uniprot database concatenated with a reverse decoy database. Trypsin was specified as a cleavage enzyme allowing 4 missing cleavages. Carbamidomethyl on Cys and oxidation on Met were specified as fixed modification and variable modification, respectively. The mass tolerance for fragment ions was set as 0.02 Da. FDR was adjusted to <1%, and the minimum score for modified peptides was 40. The proteins with more than a 1.3-fold change and those which passed the Student's *t*-test (*p* < 0.05) were selected as the differentially accumulated proteins (DAPs).

### 2.8. Bioinformatic Analysis

The Venn diagram was drawn by Venny v2.1, an online software package (https://bioinfogp.cnb.csic.es/tools/venny/index.html). Hierarchical clustering analysis was carried out using Cluster 3.0 software with the log-transformed fold induction density value in different cold acclimation treatments. A complete linkage algorithm was employed to construct the tree diagram by Treeview software (version 1.1.3). The protein-protein interaction network of DAPs was constructed by using String 11.0 (https://string-db.org) and analyzed by Cytoscape 3.5.1. The functional modules in the PPI network were identified by MCODE in Cytoscape.

### 2.9. Statistical Analysis

For morphology observations and proteomic analyses, three biological replicates were performed in the present study. Statistical significance was tested by one-way ANOVA analysis or Duncan's post-test (*p* < 0.05) for multiple comparisons with SPSS 19.0 (SPSS, Chicago, IL USA). Data in figures and tables were expressed as means ± SE.

## 3. Results

### 3.1. Morphological Observation

Compared with CK, the space of the knee joint in the KOA group was smaller (Figures 2(a) and 2(b)). However, the joint space in the AI group was bigger than that in the KOA group (Figures 2(b) and 2(c)). Moreover, the MRI results found that more fluid accumulated in the articular cavity and the surface of femoral condyle cartilage was much rougher in the KOA group than that in the CK group. On the contrary, less fluid was observed in the articular cavity and the surface of femoral condyle cartilage was smoother in the AI group than in the KOA group (Figure 3). The results of HE staining and safranin O-fast green staining showed that the surface of the cartilage was uneven and the arrangement of chondrocytes was disordered in the KOA group, but the situation was conversed in the AI group (Figure 4). Besides, several chondrocytes were tightly packed together. These results suggested that acupotomy intervention obviously alleviated the damage caused by osteoarthritis in knees.

### 3.2. Protein Identification and Differently Accumulated Protein Analysis

The changes of protein profiles in three groups were analyzed by the TMT proteome in the present study. A total of 412 differently accumulated proteins (DAPs) were identified among the three groups (data not shown). As shown in Figure 5, 132 DAPs, 100 DAPs, and 7 DAPs were specifically expressed in KOA vs. CK, AI vs. CK, and AI vs. KOA, respectively. In addition, 16 DAPs were shared by the three comparable groups.

To explore the regulatory mechanism of acupotomy intervention which alleviated KOA in rabbits, 68 DAPs in AI vs KOA are listed in Table 1. According to the protein function, these DAPs were divided into 9 groups including energy metabolism, tricarboxylic acid cycle (TCA cycle), amino acid metabolism, lipid metabolism, protein metabolism, transportation, cell development, signaling transduction, and others. The results of heatmaps of DAPs in different function groups showed that most of DAPs related to cell development and signaling transduction were increased in the AI group compared with the KOA group (Figures 6(c) and 6(h)). On the contrary, the abundances of DAPs involved in energy metabolism, the TCA cycle, amino acid metabolism, transportation, lipid metabolism and protein metabolism, and others were almost higher in the KOA group than in the IA group and CK (Figures 6(a), 6(b), 6(d)–6(g)).

### 3.3. Protein-Protein Interaction (PPI) Analyses of DAPs in AI vs. KOA

With PPI analyses, the interaction network of DAPs in AI vs. KOA was visualized in Figure 7, which contained 42 proteins and 241 edges. By using MCODE plugin in Cytoscape software, 2 clusters were isolated (Figure 8). As shown in Figure 8, there were 10 nodes with 86 edges in cluster 1 and 8 nodes with 24 edges in cluster 2, respectively. DAPs in cluster 1 were succinate dehydrogenase [ubiquinone] flavoprotein subunit (SDH1, accession: A0A5F9CIE2), oxoglutarate dehydrogenase (OGDH, accession: A0A5F9CUY0), isocitrate dehydrogenase [NAD] subunit (IDH3s, accession: G1TA59, A0A5F9D9Z6), dihydrolipoamide S-succinyltransferase (DLST, accession: A0A5F9CAW7), ATP synthase subunit alpha (ATP5F1A, accession: G1SKT4), ubiquinol-cytochrome c reductase core protein 1 (UQCRC1, accession: G1SGP1), succinate-CoA ligase subunit alpha (SUCLG1, accession: G1SKD9), acetyltransferase component of pyruvate dehydrogenase complex (DLAT, accession: G1T9S4), aconitate hydratase (ACO2, accession: G1TUX2), and succinate-CoA ligase subunit beta (SUCLA2, accession: G1U276). DAPs in cluster 2 were malate dehydrogenase (MDH2, accession: U3KMH9), solute carrier family 25 member 3 (SLC25A3, accession: G1T237), ATP synthase subunit O (ATPeF0O, accession: A0A5F9C153), cytochrome c oxidase subunit (COX6B, accession: G1SXI9), cytochrome c oxidase subunit 6A (COX6A, accession: G1ST31), cytochrome c (CYCS, accession: P00008), cytochrome c oxidase subunit 7A1 (COX7A1, accession: G1T4Q4), and cytochrome c oxidase subunit 2 (MT-CO2, accession: P98049). Based on the protein function, DAPs in cluster 1 participated in the TCA cycle (SDH1, OGDH, IDH3s, DLST, SUCLG1, DLAT, ACO2, and SUCLA2) and energy metabolism (ATP5F1A and UQCRC1). Similarly, DAPs in cluster 2 mostly participated in the TCA cycle (MDH2), energy metabolism (ATPeF0O, COX6B, COX6A, COX7A1, and MT-CO2), and transportation (SLC25A3).

## 4. Discussion

### 4.1. The Effect of Acupotomy Intervention on Knee Osteoarthritis

Knee osteoarthritis (KOA) induces a persistent abnormal load within the joint, and cartilage degeneration has always been the focus of KOA research [9–11]. The morphological observation by Safranin O staining showed that KOA causes the defect of cartilage surface and disorder of the chondrocyte arrangement, which is regarded as symptoms of cartilage degeneration [5]. Similar to the previous study, we also found that the surface of KOA cartilage was rough and the arrangement of chondrocytes was disordered (Figure 4). Moreover, the space of knee joint was smaller between KOA cartilage, which is prone to cause cartilage wearing [12, 13]. Cartilage wearing is one of main reasons for cartilage degeneration during the course of KOA. In the present study, the space of knee joints in KOA rabbits was smaller than CK, which indicated that cartilage wearing was an important reason for KOA (Figures 2 and 3).

Accumulating evidences proved that acupotomy therapy was an effective treatment for KOA [14–16]. For example, Wang et al. (2019) reported that the application of acupotomy clearly alleviated the symptoms of KOA in rabbits by changing the arrangement of fibrous tissue [8]. Besides, the application of acupotomy in rabbits significant prevented both cartilage surface erosion and subchondral bone loss by histological observation [5]. In clinical treatment, Cho et al. (2019) reported that the combined therapeutic effect of miniscalpel acupuncture and splint therapy on osteoarthritis of the hand seems to have positive results [17]. Consistent with the previous study, our results of HE staining and safranin O-fast green staining in the present study also exhibited an orderable arrangement of chondrocytes in AI (Figure 4). Moreover, several studies on acupotomy therapy revealed that acupotomy could release adhesions to alleviate the damage caused by KOA [18,19]. As shown in Figures 2 and 3, the space of knee joints was bigger in the AI group than that in the KOA group. These results were, to some extent, supported the opinion proposed by previous studies. Taken together, the morphological observation presented in our study indicated that acupotomy intervention could be an effective treatment for KOA by altering the morphology of the knee joint and the arrangement of chondrocytes. However, the mechanism of acupotomy on treating KOA was still unknown. Therefore, the proteomic analyses of acupotomy on KOA rabbits were performed in this study.

### 4.2. DAPs Related to Energy Metabolism and TCA Cycle

As the main subcellular organelles to produce energy in cells, mitochondria control the conversion of energy and primary metabolites by various biological processes, such as glycolysis, the TCA cycle, the oxidative phosphorylation system, and so on [20]. Previous studies found that mitochondrial function was tightly associated with osteoarthritis pathophysiology [21, 22]. Moreover, some evidences showed that osteoarthritis induced the energy production in chondrocytes [21, 23, 24]. In other words, more energy production was a symptom of osteoarthritis in chondrocytes. Similar to previous studies, we also found that DAPs related to energy metabolism were mostly up-regulated in KOA compared with CK (Figure 6(a), Table 1). However, AI treatment reduced the abundances of these DAPs (Figure 6(a), Table 1). For example, the subunits of cytochrome c oxidase (complex IV) and cytochrome b-c 1 complex (complex III), which are the main components of respiratory chain to product energy in mitochondria [22], were firstly up-regulated in KOA vs. CK but down-regulated in AI vs. KOA (Figure 6(a), Table 1). Furthermore, we found that the ATPase inhibitor (ATP5IF1, assession: G1TES2) exhibited a reverse trend compared with DAPs related to cytochrome c oxidase. ATP5IF1 was proved to function as a regulator to avoid the consumption of cellular ATP [25]. The accumulation of ATP5IF1 in AI vs. KOA but degradation in KOA vs. CK indicated that ATP5IF1 might function as a crucial regulator induced by AI to balance the energy synthesis and consumption in chondrocytes of rabbits. Besides, the TCA cycle was found to play a central role in energy production in osteoarthritis chondrocytes by changing the central metabolism [21, 24]. In the present study, 11 DAPs involved in the TCA cycle were totally up-regulated in KOA vs. CK but down-regulated in AI vs. KOA (Figure 6(b)). Based on these results, it was suggested that KOA promoted the accumulation of proteins related to energy metabolism and the TCA cycle but down-regulated of ATP5IF1 to product more energy as an immune response of KOA, while AI alleviated KOA by reducing the accumulation of proteins related to energy metabolism and the TCA cycle but up-regulated ATP5IF1 to limit the energy consumption. Furthermore, our PPI analyses found that most of DAPs in cluster1 and cluster 2, which were the core subnetwork isolated from the whole PPI network, were involved in the TCA cycle and energy metabolism, which implied that DAPs related to the TCA cycle and energy metabolism play a central role in response to KOA and AI (Figures 7 and 8).

### 4.3. DAPs Related to Cell Development

As shown in Figure 6, DAPs related to cell development were totally up-regulated, such as fibronectin (FN1, accession: A0A5F9CPW4), vimentin (VIM, accession: G1SWS9), collagen (COL12A1, COL14A1, accession: A0A5F9D4Y9, A0A5F9DVP3), myosin (MYBPH, accession: G1T0G2), and dihydropyrimidinase like 3 (DPYSL3, accession: A0A5F9CLG7). A recent study reported that fibronectin significantly promoted cartilage repair by enhancing the proliferation, migration, and chondrogenic differentiation of chondrogenic progenitor cells [26]. The stimulation of the regenerating endogenous cells was considered a novel cartilage repair strategy during KOA treatment [26]. As FN1 was up-regulated after the operation of AI, it was suggested that AI could be an available treatment to alleviate KOA by promoting the synthesis of fibronectin to repair the damaged cartilage tissue. As a main component of chondrocyte cytoskeleton, vimentin played an important role in maintaining the stiffness of chondrocytes in osteoarthritis [27]. In addition, dihydropyrimidinase-related protein 1, which is a homologous protein with dihydropyrimidinase-like 3, was proved to have participated in remodelling of the cytoskeleton in human cells [28]. Similarly, collagen is a structural component of many musculoskeletal tissues, and the inhibition of collagen synthesis would result in cartilage damage [29]. Particia et al. (2018) suggested that enhancing collagen synthesis could help the regeneration of cartilage, which could be a treatment of osteoarthritis [30]. In our proteomic data, the accumulation of collagen, vimentin, and dihydropyrimidinase-like 3 in AI vs KOA indicated that AI could alleviate KOA by maintaining the stiffness of chondrocytes and promoting the regeneration of cartilage. Besides, muscle weakness is also a major clinic symptom of osteoarthritis. In rats, the application of caicalin could attenuate the dysfunction of muscles in OA rats by promoting the expression of myosin [31]. In other words, the accumulation of myosin might have a protective effect in muscles that suffered from OA. Consistent with the previous study, in the present study, the fact that DAPs related to myosin were up-regulated in AI vs. KOA implied that AI could attenuate KOA by enhancing the expression of myosin. Based on these literature studies and our proteomic results, we suggested that AI-induced FN1, VIM, COL12A1, COL14A1, MYBPH, and DPYSL3 played important roles in the treatment of KOA.

### 4.4. DAPs Related to Signaling Transduction

Protein histidine methylation is a new-typepost-translational modification, which is catalyzed by protein-histidineN-methyltransferase [32]. In vitro, histidine N-methyltransferase (SETD3) was found to function in regulating the methylation at beta-actin H73, which affected the synthesis of cellular F-actin and the glycolytic phenotype [32], and actin or the actin pathway in chondrocytes was proved to control both skeletal development and associated diseases such as osteoarthritis [33]. As protein-histidineN-methyltransferase (SETD3, accession: A0A5F9DM36) was up-regulated in KOA rabbits after the operation of AI, we speculated that AI could alleviate KOA in chondrocytes by regulating methylation of actin mediated by SETD3.

Cyclophilin B (CyPB), encoded by peptidyl-prolylcis-trans isomerase (PPIB), was proposed to indirectly regulate the hydroxylation of collagen and impact collagen glycosylation and fibrillogenesis [34]. Collagen hydroxylation was found to be an important process in cartilage healing [35]. In this study, the abundance of peptidyl-prolylcis-trans isomerase (PPIB, accession: G1T2F2) increased in AI but did not change in KOA which implied that AI-induced PPIB might function as a key regulator in KOA healing by controlling the hydroxylation of collagen and fibrillogenesis.

Apoptosis-inducing factor mitochondrial associated 1 (AIFM1, accession: U3KP10) functions not only as a regulator of apoptosis but also as a regulator of respiratory chain biogenesis [36]. In AIF-deficient cells, the respiratory function was reduced, but it could be reestablished by CHCHD4, which is an AIF-interacting protein to control the import of various metabolites [36]. Respiratory chain is the major biological process to produce energy in mitochondria. In this study, the abundance of AIFM1 was increased in KOA but reduced in AI, which was consistent with the change of DAPs related to energy metabolism and TCA cycle, and this indicated that AIFM1 was an important regulator in mitochondria to control the energy production, such as the TCA cycle.

## 5. Conclusion

The mechanism of acupotomy intervention (AI) on the treatment of knee osteoarthritis (KOA) was investigated in this study. The results of morphological observations indicated that AI alleviated KOA by altering the morphology of the knee joint and the arrangement of chondrocytes. With proteomic analyses, 68 differently accumulated proteins (DAPs) were identified in AI vs. KOA and divided into 9 groups. With protein-protein interaction analyses, DAPs related to energy metabolism and the TCA cycle were suggested to play a central role in response to AI. Moreover, AIFM1 was proposed to be an important regulator in controlling the energy production in mitochondria. In addition, DAPs involved in cell development, such as FN1, VIM, COL12A1, COL14A1, MYBPH, and DPYSL3, might function as AI-responsive proteins, which were important for the treatment of KOA.

## Figures and Tables

**Figure 1:** The diagram for TMT proteomic analysis from protein extraction to bioinformatic analysis.

**Figure 2:** The X-ray images of rabbit's left knee among different treatments. (a) CK represents control, (b) KOA represents rabbits with knee osteoarthritis, and (c) AI represents KOA rabbits treated with acupotomy intervention. Compared with CK, the space between knee joints in KOA rabbits was smaller, but the knee joint space in the AI group was similar to that in CK.

**Figure 3:** The MRI images of rabbit's knee joints among different treatments. (a), (b), and (c) were the sagittal section of the knee joint; (d), (e), and (f) were the comal plane of the knee joint. The red arrow in (b) showed that the knee joint space in the KOA group was much smaller than that in the other two groups. The red arrows in (e) showed that the surface of femoral condyle cartilage was somewhat rough.

**Figure 4:** The histomorphological observation of femoral condyle cartilage in three treatments by HE staining and safranin O-fast green staining. (a), (b), and (c) were the images of femoral condyle cartilage stained by HE. (d), (e), and (f) were the images of femoral condyle cartilage by safranin O-fast green staining.

**Figure 5:** The Venn diagram analysis of DAPs among CK, KOA, and AI groups.

**Figure 6:** Hierarchical clustering analysis of the differentially accumulated proteins (DAPs) in CK, KOA, and AI treatments. (a) Energy metabolism, (b) the TCA cycle, (c) cell development, (d) amino acid metabolism, (e) transportation, (f) lipid metabolism, (g) protein metabolism and others, and (h) signaling transduction. The intensity of the color represents the abundance of protein shown at the right bottom.

**Figure 7:** The protein-protein interaction network of DAPs in AI vs. KOA.

**Figure 8:** The clustering analysis of PPI network in AI vs. KOA. (a) Cluster 1 containing 10 nodes and 86 edges, while cluster 2 containing 8 nodes and 24 edges.

**Table 1:** The information of differently accumulated proteins (fold change <0.7 or >1.3) in the acupotomy intervention (AI) group vs. the knee osteoarthritis (KOA) group.

Accession	Protein description	Gene name	MW (kDa)	Coverage (%)	Peptides	Ratio	*p* value
Energy metabolism							
G1T0U9	Creatine kinase S-type, mitochondrial	CKMT2	47.45	38.70	14	0.50	0.0124
G1SZ23	3-Hydroxybutyrate dehydrogenase 1	BDH1	37.69	11.40	4	0.58	0.0012
G1SXI9	Cytochrome c oxidase subunit	COX6B	10.17	47.70	4	0.59	0.0147
G1T4Q4	Cytochrome c oxidase subunit 7A1	COX7A1	8.87	16.50	1	0.63	0.0183
G1TZN7	Cytochrome c oxidase subunit 5A	COX5A	20.42	23.60	3	0.65	0.0213
G1TCZ0	Cytochrome c oxidase subunit 5B	COX5B	13.76	24.80	3	0.68	0.0475
G1SG11	Cytochrome c oxidase subunit 4 isoform 1, mitochondrial	COX4I1	19.55	26.00	4	0.69	0.0475
U3KMU6	Cytochrome b-c1 complex subunit Rieske, mitochondria	UQCRFS1	14.95	10.40	1	0.65	0.0283
P98049	Cytochrome c oxidase subunit 2	MT-CO2	25.97	15.90	3	0.71	0.0231
G1ST31	Cytochrome c oxidase subunit 6A, mitochondrial	COX6A	14.72	17.30	2	0.65	0.0439
A0A5F9CAY2	Cytochrome c oxidase subunit 4 isoform 1, mitochondrial	COX4I1	10.04	20.50	1	1.54	0.0016
G1SDJ3	ATP synthase membrane subunit DAPIT	DAPIT	6.42	25.90	1	0.60	0.0311
A0A5F9C153	ATP synthase subunit O, mitochondrial	ATPeF0O	25.72	32.90	6	0.73	0.0370
G1SKT4	ATP synthase subunit alpha	ATP5F1A	59.75	28.60	14	0.75	0.0433
G1T9N2	ATP synthase subunit d, mitochondrial isoform X2	ATPeF0D	15.74	24.80	3	0.77	0.0376
G1TES2	ATPase inhibitor, mitochondrial	ATP5IF1	16.77	12.80	2	4.18	0.0054
U3KNE2	NDUFA4, mitochondrial complex-associated	NDUFA4	9.33	37.80	3	0.65	0.0078
A0A5F9DDY7	UQCRC2 isoform 4	QCR2	44.51	35.40	10	0.68	0.0370
G1SGP1	Ubiquinol-cytochrome c reductase core protein 1	UQCRC1	52.41	31.90	11	0.72	0.0237
A0A5F9DAA7	Thioredoxin domain-containing protein	PRDX3	30.15	19.80	5	0.73	0.0059
TCA cycle							
U3KMH9	Malate dehydrogenase	MDH2	40.53	37.00	11	0.62	0.0322
G1SKD9	Succinate--CoA ligase subunit alpha, mitochondrial	SUCLG1	36.22	13.30	4	0.63	0.0330
G1U276	Succinate--CoA ligase subunit beta, mitochondrial	SUCLA2	58.44	24.60	12	0.64	0.0142
A0A5F9CIE2	Succinate dehydrogenase [ubiquinone] flavoprotein subunit	SDH1	60.33	15.00	7	0.69	0.0231
G1TA59	Isocitrate dehydrogenase [NAD] subunit, mitochondrial	IDH3A	49.04	11.00	4	0.64	0.0137
A0A5F9D9Z6	Isocitrate dehydrogenase [NAD] subunit, mitochondrial	IDH3B	40.96	14.40	4	0.74	0.0108
G1TUX2	Aconitate hydratase, mitochondrial	ACO2	87.35	33.10	20	0.69	0.0388
G1T9S4	Acetyltransferase component of pyruvate dehydrogenase complex	DLAT	68.20	8.70	5	0.71	0.0383
A0A5F9DJY5	Pyruvate dehydrogenase E1 alpha 1 subunit	PDHA1	40.17	29.20	10	0.74	0.0299
A0A5F9CUY0	Oxoglutarate dehydrogenase	OGDH	113.61	23.80	21	0.75	0.0206
A0A5F9CAW7	Dihydrolipoamide S-succinyltransferase	DLST	48.58	25.30	8	0.76	0.0329
Amino acid metabolism							
G1SW97	Isovaleryl-CoA dehydrogenase	IVD	46.31	9.90	4	0.69	0.0407
A0A5F9DQB1	3-Hydroxyisobutyrate dehydrogenase	HIBADH	34.27	5.80	1	0.67	0.0250
A0A5F9DH24	Aminoadipate-semialdehyde synthase	AASS	96.45	3.80	3	0.74	0.0240
G1SP32	3-Hydroxyisobutyryl-CoA hydrolase, mitochondrial	HIBCH	43.43	8.00	3	0.75	0.0053
P00008	Cytochrome c	CYCS	11.69	21.00	3	0.62	0.0461
Lipid metabolism							
G1U891	HADHB isoform 1	HADHB	49.74	17.80	7	0.68	0.0405
G1SCE7	HADHB isoform 1	HADHB	51.45	19.20	8	0.73	0.0124
G1SPY9	Acyl-CoA synthetase medium chain family member 5	ACSM5	64.60	5.50	3	0.73	0.0363
G1SPZ9	Pyrophosphatase (inorganic) 2	PPA2	38.73	8.80	2	0.76	0.0241
G1SRD2	KAT8 regulatory NSL complex subunit 1 like	KANSL1L	44.04	16.70	5	0.71	0.0363
Protein metabolism							
A0A5F9CND9	R3H domain-containing 1	R3HDM1	111.07	1.30	1	0.74	0.0415
G1SI29	Elongation factor tu	TUFM	49.71	17.80	6	0.76	0.0325
U3KLZ3	Heterogeneous nuclear ribonucleoprotein A3	HNRNPA1	37.67	9.00	3	1.39	0.0310
Transportation							
G1SER3	Solute carrier family 25 member 11	SLC25A11	34.06	18.20	5	0.62	0.0195
G1T2J6	Solute carrier family 25 member 12	SLC25A12	71.46	14.30	9	0.70	0.0459
G1T237	Solute carrier family 25 member 3	SLC25A3	39.90	13.00	4	0.73	0.0326
P12345	Aspartate aminotransferase, mitochondrial	GOT2	47.41	23.30	9	0.62	0.0463
G1T332	Aspartate aminotransferase	GOT1	46.46	21.30	8	0.63	0.0126
G1SG30	NipSnap homolog 2	NIPSNAP2	30.64	19.10	4	0.64	0.0319
O46373	ADP/ATP translocase 1	SLC25A4	32.90	26.80	8	0.68	0.0390
P68003	Voltage-dependentanion-selective channel protein 2	VDAC2	31.58	31.60	7	0.72	0.0444
Cell development							
Q95MN6	Proteolipid protein 2	PLP2	16.75	8.60	1	1.31	0.0130
A0A5F9CPW4	Fibronectin	FN1	226.97	2.10	3	1.37	0.0020
G1SWS9	Vimentin	VIM	53.65	44.40	20	1.48	0.0219
A0A5F9D4Y9	Collagen alpha-1(XII) chain	COL12A1	203.08	1.60	3	1.59	0.0445
G1T0G2	Myosin binding protein H	MYBPH	54.31	31.40	13	1.60	0.0170
A0A5F9DVP3	Collagen type XIV alpha 1 chain	COL14A1	181.26	16.50	23	1.64	0.0220
A0A5F9CLG7	Dihydropyrimidinase like 3	DPYSL3	62.50	3.00	2	1.96	0.0379
G1SNE8	S_100 domain-containing protein	S100A10	21.97	14.10	3	1.36	0.0245
Signaling transduction							
A0A5F9CM55	Myosin heavy chain 2	MYH	79.94	50.60	39	0.74	0.0484
U3KP10	Apoptosis inducing factor mitochondria associated 1	AIFM1	66.16	14.10	7	0.66	0.0191
A0A5F9DM36	Protein-histidineN-methyltransferase	SETD3	66.55	3.70	2	1.31	0.0192
G1T2F2	Peptidyl-prolylcis-trans isomerase	PPIB	24.06	6.00	1	1.33	0.0311
G1U0N7	Olfactory receptor family 10 subfamily J member 3	OR10J3	34.81	4.80	1	1.43	0.0375
A0A5F9CI92	Reverse transcriptase domain-containing protein	CSMD	45.89	3.20	1	1.91	0.0491
Others							
G1TRK3	Morphine-6-dehydrogenase	PGER4	36.48	22.90	5	1.36	0.0246
G1T641	4HBT domain-containing protein	ACOT13	41.43	8.10	3	0.66	0.0149

## Data Availability

The data presented in this study are available in the article.

## Abbreviations

ACO2: Aconitate hydratase
AI: Accupotomy intervention
AIFM1: Apoptosis inducing factor mitochondria associated 1
ATP5F1A: ATP synthase subunit alpha
ATPeF0O: ATP synthase subunit O
BCA kit: Bicinchoninic acid assay kit
COL12A1: Collagen alpha-1(XII) chain
COL14A1: Collagen type XIV alpha 1 chain
COX6B: Cytochrome c oxidase subunit
COX6A: Cytochrome c oxidase subunit 6A
COX7A1: Cytochrome c oxidase subunit 7A1
CYCS: Cytochrome c
CyPB: Cyclophilin B
DAP: Differently accumulated proteins
DLAT: Acetyltransferase component of pyruvate dehydrogenase complex
DLST: Dihydrolipoamide S-succinyltransferase
DPYSL3: Dihydropyrimidinase like 3
FN1: Fibronectin
HE: Hematoxylin-eosin
IDH3s: Isocitrate dehydrogenase [NAD] subunit
KOA: Knee osteoarthritis
LC-MS/MS: Liquid chromatograph-mass spectrometer/mass spectrometer
MDH2: Malate dehydrogenase
MRI: Magnetic resonance imaging
MT-CO2: Cytochrome c oxidase subunit 2
MYBPH: Myosin binding protein H
OGDH: Oxoglutarate dehydrogenase
PPI: Protein-protein interaction (PPI)
PPIB: Peptidy-prolyl cis-trans isomerase
SDH1: Succinate dehydrogenase [ubiquinone] flavoprotein subunit
SUCLG1: Succinate-CoA ligase subunit alpha
SUCLA2: Succinate-CoA ligase subunit beta
SLC25A3: Solute carrier family 25 member 3
SETD3: Histidine N-methyltransferase
TMT: Tandem mass tags
TCM: Traditional Chinese medicine: TCM
TEAB: Tetraethyl ammonium bromide
TCA cycle: Tricarboxylic acid cycle
VIM: Vimentin
UPLC: Ultra high performance liquid chromatography
UQCRC1: Ubiquinol-cytochrome c reductase core protein 1.
